The article "Genetic Programming-Based Feature Selection for Emotion Classification Using EEG Signal" was published in 2022. Journal: J Healthc Eng.

# Genetic Programming-Based Feature Selection for Emotion Classification Using EEG Signal

**DOI:** 10.1155/2022/8362091

**Published:** 2022-03-08

**Authors:** Aditi Sakalle, Pradeep Tomar, Harshit Bhardwaj, Asif Iqbal, Maneesha Sakalle, Arpit Bhardwaj, Wubshet Ibrahim

**Affiliations:** ^1^CSE Department, University School of Information and Communication Technology, Gautam Buddha University, Greater Noida, India; ^2^SDITS College of Engineering, Khandwa, India; ^3^Department of Mathematics, SNGPG, College Khandwa, Khandwa, India; ^4^CSE Department, BML Munjal University, Haryana, India; ^5^Department of Mathematics, Ambo University, Ambo, Ethiopia

## Abstract

The COVID-19 has resulted in one of the world's most significant worldwide lock-downs, affecting human mental health. Therefore, emotion recognition is becoming one of the essential research areas among various world researchers. Treatment that is efficacious and diagnosed early for negative emotions is the only way to save people from mental health problems. Genetic programming, a very important research area of artificial intelligence, proves its potential in almost every field. Therefore, in this study, a genetic program-based feature selection (FSGP) technique is proposed. A fourteen-channel EEG device gives 70 features for the input brain signal; with the help of GP, all the irrelevant and redundant features are separated, and 32 relevant features are selected. The proposed model achieves a classification accuracy of 85% that outmatches other prior works.

## 1. Introduction

Due to the COVID-19 epidemic, all the governments in the world have to impose a lockdown. This strictness, however, affects the emotions of the people, and lots of people are feeling emotional imbalance [1]. The people are experiencing negative emotions, and their health and performance are degrading day by day. Emotion and mental awarenesses have become the primary concern for all the governments in the world because a lot of people are feeling stressed and alone [2].

To address the challenge as mentioned above, lots of researchers are applying classification algorithms to understand the emotion of the people [3]. Humans cannot classify these types of emotions; whereas, these classifiers can do this task very efficiently [4]. Recently, many expert systems and machine learning tools are gaining importance for the classification of medical data because they can learn from experience, past patterns, and examples [5–7]. Also, a more detailed medical data examination can be done in a shorter time with a reduced number of errors [8–10]. However, the problem with many features is that they are redundant. Because of that, they increase the error rather than reducing it [11, 12]. Feature selection can address this problem by selecting only relevant features for classification [13–15]. This improves the performance of the classifiers by removing similar features, shortening the training time. The techniques like evolutionary algorithms are gaining importance in feature selection because they can efficiently search the entire search space. There are few evolutionary algorithms, but genetic programming has shown good results on classification problems. Another advantage of using GP is that the classifier of GP has a tree structure [16], so we can recognize the features present in the best classifier. This will help, especially in the case of medical diagnosis, because we can determine which features are more important. In the last decade, there have been several reports on applying GP techniques to a range of medical data classification problems [17–19].

The article "Genetic Programming-Based Feature Selection for Emotion Classification Using EEG Signal" was published in 2022. Journal: J Healthc Eng.

However, in this study, the genetic programming-based feature selection (FSGP) technique is proposed. It helps to improve the classification accuracy of the emotion recognition dataset by removing redundant and irrelevant characteristics in a single GP life cycle. An EEG dataset is created using brain signals [20]. The proposed algorithm yielded an accuracy of 85% for 80–20 training-testing partition. The results show that our approach works well with the EEG database and reduces the number of features with increased classification accuracy, confirming that it can be an excellent alternative to the well-known expert system and machine learning methods. The goal of our algorithm would be to correctly classify the samples as positive and negative emotions with an optimal number of features. The following few points highlight the difference between the current study and the existing ones in the literature. (i) How we can reduce the number of features and simultaneously increase the classification accuracy in a single genetic programming life cycle. (ii) The present study contains the result on the emotion recognition dataset created using the 14-channel EEG device. (iii) A reduced number of features are also presented along with the classification accuracy.

The rest of the study is described as follows: Section 2 gives the device and dataset description, Section 3 tells about the proposed algorithm, Section 4 presents the result of the proposed algorithm, and Section 5 compares the proposed algorithm with other machine learning algorithms.

## 2. Methods and Materials

This part provides information about the device, dataset used, and the classification algorithm.

### 2.1. Device Description

Emotiv EPOC is a 14-channel wireless headband for collecting brain signals shown in Figure 1. It is a portable device that has 14 electrodes following the American EEG Society Standard, as shown in Figure 2. This device can collect raw EEG data and generate the features from the signals. The total number of signals this device generates is 70. The five features are from every 14 channels, so 70 features.

The article "Genetic Programming-Based Feature Selection for Emotion Classification Using EEG Signal" was published in 2022. Journal: J Healthc Eng.

The EEG signals are generated as a person experiences different emotions or feelings when exposed to situations or scenarios through visual content. We recognize an individual's emotions by analyzing brain waves while watching emotional or situational materials and classify the emotions into two classes, i.e., positive and negative. The elicitation materials included around 60 videos, which depict the dramatic person's predefined personality traits and are therefore recognized as the ground truth of this work's experimental procedure.

### 2.2. Dataset

Fifty (25 males and 25 females) nonclinical participants were considered for this research. The study was volunteered by participants, and an informed consent form was also concluded. All nonclinical participants from various cultures and education classes were Hindi speaking. However, 5 data samples were dropped as a result of failure in equipment or excessive EEG signal artifacts in the final analysis. The age group of participants is divided into three age groups as 15–20 years, 21–26 years, and 27–35 years.

## 3. Proposed Method

For this research, fifty (25 males and 25 females) nonclinical participants involved. Participants volunteered for the study, and an informed consent form was also concluded—all nonclinical participants from various cultures and education classes were Hindi speaking. However, 5 data samples were dropped due to failure in equipment or excessive EEG signal artifacts in the final analysis; in total, 45 participants were considered for this research. 

### 3.1. Initialization and Fitness

We generate the initial population using all features in the feature set and terminals in the terminal set. The ramped half and half method is used for initializing the population. We maintain the structural diversity of the people through all generations. To keep the variety, all the individuals are compared to ensure that no similar trees are generated. After generating the diverse initial population, we calculate the fitness of all the trees using the emotion recognition dataset. During training the individuals, we calculate the fitness using the training dataset.

### 3.2. Feature Selection

After evaluating the fitness of the classifiers, we perform our feature selection process. In this, we calculate the average fitness of the classifiers in the generation. After that, we select those classifiers whose accuracy (fitness) is more significant than average accuracy and named them Cgaa classifiers (classifier having accuracy greater than average accuracy). Then, we assign the weights to the features present in Cgaa classifiers. Initially, the weight of all the features is 0; then, we evaluate the number of times any feature is present in these Cgaa classifiers. The number of times the feature is present in the Cgaa classifier is the weight of that feature. This process is repeated for all the features, and their weights are evaluated. We repeat this process for 50% of the generation and evaluate the weight of all the features present in Cgaa classifiers. After getting the weight of all the features, we calculate their average. Those features whose weights are more significant than average weight is selected, and we named them suboptimal features (Fso). Then, we got two subsets of features: those whose weight is more significant than average weight (Fso) and those whose weight is not greater (Fno).

The article "Genetic Programming-Based Feature Selection for Emotion Classification Using EEG Signal" was published in 2022. Journal: J Healthc Eng.

In the next generation, we replace all the (Fno) features with (Fso) features. To replace the (Fno) features with (Fso) features, we apply a modified mutation technique, in which we replace the single (Fno) feature with a single (Fso) feature randomly chosen from the (Fso) subset. Then, we compare the fitness of the newly generated tree with its parent. If the fitness of the tree is increased, then we stop; otherwise, we repeat this process till we get better offspring than a parent. In this way, all the unwanted (Fno) features are replaced by (Fso) features. Then, we allowed the GP life cycle to run till the last generation and obtain the best classifier in terms of fitness, and the features present in the best classifier are the optimal feature set. The advantage of this method is that we had done the feature selection and classification in one run of GP. The other benefit is that our process does not suffer from overfitting problems as happens in the case of wrapper approaches because of applying a similar algorithm two times, the first time for feature selection and the second time for classification. The flowchart of the proposed work is shown in Figure 3.

### 3.3. Genetic Operators

The three operators of genetic programming are applied to generate the following populations. Reproduction copies the best individual to the next generation. Crossover and mutation operators are improved to reduce the possibility of sending the lower fitness individuals to the next generations. The hill-climbing crossover and mutation operators [16] are used in this work. After doing the crossover and mutation, the offsprings are compared with their parents, and if their fitness is better than the parents, only the child is transferred to the next generation. Due to this property only, the exploitation of the solution is maintained.

The article "Genetic Programming-Based Feature Selection for Emotion Classification Using EEG Signal" was published in 2022. Journal: J Healthc Eng.

### 3.4. Termination Criteria

The GP process is terminated as soon as the fitness reaches 100% accuracy.

## 4. Results

In this section, the FSGP model results are examined. The computer configuration consists of 64 GB RAM-based Python (3.8) for incorporating FSGP, GPmtfs, and another existing approaches, i.e., neural network, genetic programming, random forest, and SVM. These algorithms were applied to the EEG dataset for emotion recognition. Experimentation is carried out on the datasets with the parameters as given in Table 1.

In this study, the dataset is separated into two parts, i.e., in training and test sets. They are divided into different partitions to compare the training-testing outcomes to existing literature.

The performance assessment is conducted using a hold-out 80–20 validation scheme. In the 80–20 partition scheme, we have divided the dataset into two parts; the first part consists of 80%, which is used for training the model and the second part consisting of 20% is for model testing. The proposed FSGP and GPmtfs architecture were evaluated by calculating the performance metrics such as sensitivity, precision, and specificity values and are given in Table 2, and their mathematical expressions are given as follows.

(1) $$\begin{array}{c} \text{Recall}=\frac{TP}{TP+FN}\\ \text{Precision}=\frac{TP}{TP+FP}\\ \text{Specificity}=\frac{TN}{TN+FP}. \end{array}$$

where TP is true positive, TN is true negative, FP is false positive, and FN is false negative.

In this section, we present the experimental results to test the behavior of the proposed genetic programming-based feature selection (FSGP) model, as well as to compare it with the classical multitree genetic programming-based FS (GPmtfs) model [14]. The results of classification accuracy of both the models are given in Table 3, with 80–20 training and testing data for the emotion recognition dataset. It is clear from the results that the FSGP model outperforms the classical GPmtfs in terms of classification accuracy for 80–20 training-testing data. It is also clear from the result that the average number of features selected by the FSGP model is less than the GPmtfs model, which shows that replacing the unwanted features in the middle stage with suboptimal features helps select the optimal set of features and improves the accuracy. Classification accuracy achieved by the FSGP model for 80–20 training-testing samples is 85% with 32 average number of features for the EEG dataset, which is very remarkable. It shows that the FSGP model has good adaptation generation capability and can select the optimal number of features if proper training data are provided. The result confirms the importance of appropriate training data for selecting the optimal features from the dataset.

The article "Genetic Programming-Based Feature Selection for Emotion Classification Using EEG Signal" was published in 2022. Journal: J Healthc Eng.

This concludes that our FSGP can reduce the number of features with improved accuracy and show the important features in the dataset. Thus, our model can be a beneficial tool for physicians to diagnose the patient.

The GPmtfs model' maximum, average, and minimum classification accuracies for 80–20 training-testing partition achieved are 75%, 71%, and 68%, respectively.

The FSGP model' maximum, average, and minimum classification accuracies for 80–20 training-testing partition achieved are 85%, 82%, and 80%, respectively.

Table 4 provides the accuracy of the FSGP model on a different number of fitness evaluations. It is clear from the results that the model gives the best accuracy at 80000 fitness evaluations. The accuracy below those numbers is inferior, and after 80000 fitness evaluation, the accuracy is not improving. This suggests that our model converges at 80000 fitness evaluations.

Figure 4 shows the comparison of the accuracy of GPmtfs and FSGP on a different number of evaluations. Both algorithms do not seem to produce good results when the number of fitness evaluations is less. On increasing the fitness evaluations, the accuracy of both models increases; however, FSGP outperforms GPmtfs on every comparison. Both the models converged around 80000 fitness evaluations and marked their complete accuracy.

Figure 5 shows the accuracy and features of the FSGP model on a different number of fitness evaluations. The red line indicates the accuracy, and the blue line shows the features. It is clear from the figure that the FSGP model has the highest accuracy and the lowest features at 80000 fitness evaluations. The optimal number of fitness evaluations for the FSGP model is 80000 for emotion recognition data. This fitness evaluation gives the highest accuracy with an optimal number of features.

Table 5 provides the classification accuracy in the form of confusion matrix. It is clear from Table 5 that the sum of true positive and true negative is much better for FSGP as compared to GPmtfs. This again confirms the superiority of FSGP over GPmtfs. The Mann–Whitney confirms the statistical difference in result given in Table 6. The solution produced by our FSGP model is statistically different from the GPmtfs model for 80–20 training-testing partition for the emotion recognition dataset.

## 5. Discussion

This section compares the proposed model with the standard machine learning algorithms. The conventional algorithms are also implemented using the same set of EEG features used to develop the proposed model.  Table 7 provides the classification accuracy comparison of the proposed models on the 80–20 partition scheme.

The article "Genetic Programming-Based Feature Selection for Emotion Classification Using EEG Signal" was published in 2022. Journal: J Healthc Eng.

### 5.1. Comparison

Various works from different authors on emotion recognition datasets are given in Table 7. Our proposed approach, FSGP, in which we have simultaneously done the feature selection and classification, is noteworthy in terms of classification accuracy than other approaches. Observations also show that our method removes the redundant and irrelevant features and finds the optimal number of features to classify the emotion recognition data.

The neural network, random forest, genetic programming, and SVM are the other state-of-the-art approaches used. To guarantee that the conclusions and comparisons given are explicit and accurate, the setting of parameters for all these classifiers has been implemented using the same method. It is evident from Table 7 that in the FSGP model, the classification accuracy was superior to all the other models for 80–20 training-testing partition. The second-best classification accuracy after FSGP is of genetic programming, and for the 80–20 training-test partition, the overall accuracy is 79%. Table 2 provides the values of FSGP and GPmtfs for 80–20 data partitioning scheme for sensitivity, precision, and specificity. It is clear from the result that FSGP outperforms the GPmtfs in all aspects.

Table 6provides the two-tailed Mann–Whitney test which shows the statistical result disparity [21]. The *p* value is computed using the Mann–Whitney test. If the *p* value is more significant than 0.05, the results do not alter considerably; nevertheless, if the *p* value is smaller than the value 0.001, the results are highly effective. The findings in Table 6 show that FSGP model results are statistically separate from GPmtfs for the 80–20 training-testing split. The results show a significant difference when these classifiers' *p* values are compared to FSGP. According to the evaluation findings, the suggested FSGP model for performance analysis of two classes of emotion, i.e., positive and negative classification, produces accurate output.

## 6. Conclusion

A novel approach for emotion recognition has been explored to extract important features and improve accuracy. This is done by removing the redundant and irrelevant features during 50% of the generation and forming a subset of suboptimal features rather than finding the optimal features that increase the classifier's accuracy after complete generation. Several experiments have been conducted with the proposed method, and a comparison has been presented with the classical GPmtfs model. The collected EEG dataset was used in this study.

The article "Genetic Programming-Based Feature Selection for Emotion Classification Using EEG Signal" was published in 2022. Journal: J Healthc Eng.

## Figures and Tables

**Figure 1:** 14-channel Emotiv EPOC.

**Figure 2:** American Society Standard for putting 14-channel electrodes.

**Figure 3:** Flowchart of the proposed work.

**Figure 4:** Accuracy of GPmtfs and FSGP on different fitness evaluations.

**Figure 5:** Accuracy of FSGP with features on different fitness evaluations.

**Table 1:** Parameter and values for the GP model.

Parameter	Value
Crossover probability	60%
Reproduction probability	20%
Mutation probability	20%
Population size	100
Initialization method	Ramped half and half
Initial maximum depth of a tree	10
Initial minimum depth of a tree	5

**Table 2:** Comparison of performance measures.

Method	Sensitivity (%)	Precision (%)	Specificity (%)
	Mean ± std	Mean ± std	Mean ± std
GPmtfs	**70.29 ± 3.16**	**78.50 ± 3.42**	76.47 ± 2.36
FSGP	**84.29 ± 1.16**	**86.50 ± 1.42**	87.47 ± 2.36

Bold shows the maximum values.

**Table 3:** Classification accuracy comparison of GPmtfs and FSGP models for the emotion recognition dataset.

Method	No. of features	Accuracy		
		Max	Avg	Min
GPmtfs	42	75	71	68
FSGP	32	85	82	80

**Table 4:** FSGP model accuracy on different numbers of fitness evaluations.

Number of fitness evaluations	Accuracy (%)
50000	66
60000	68
70000	75
80000	85
90000	84
100000	84

**Table 5:** Confusion matrix of GPmtfs and FSGP models for the emotion recognition dataset.

	GPmtfs		FSGP	
	FP	FN	FP	FN
TP	42	75	71	68
TN	32	85	82	80

**Table 6:** *P* value for FSGP.

Method	Partition	*P* value
FSGP	70–30	2.871 × 10^−11^

**Table 7:** Classification accuracy comparison of existing approaches and MLSTM_3 classifier for two class of emotion classification to analyze the mental state during pandemic.

Method	Partition	Accuracy (%)
		Max
Neural network	80–20	74
Random forest	80–20	70
Genetic programming	80–20	79
SVM	80–20	76
FSGP	80–20	**85**

Bold shows the maximum value of accuracy.

## Data Availability

The data used to support the findings of this are available from the corresponding author upon request.

## References

[1] Holmes E. A., O’Connor R. C., Perry V. H. (2020). Multidisciplinary research priorities for the covid-19 pandemic: a call for action for mental health science. *The Lancet Psychiatry*.

[2] Ren Y., Qian W., Li Z. (2020). Public mental health under the long-term influence of covid-19 in China: geographical and temporal distribution. *Journal of Affective Disorders*.

[3] Gao Y., Lee H. J., Mehmood R. M. Deep learninig of eeg signals for emotion recognition.

[4] Li R., Ren C., Zhang X., Hu B. (2022). A novel ensemble learning method using multiple objective particle swarm optimization for subject-independent eeg-based emotion recognition. *Computers in Biology and Medicine*.

The article "Genetic Programming-Based Feature Selection for Emotion Classification Using EEG Signal" was published in 2022. Journal: J Healthc Eng.

[5] Si T., Bagchi J., Miranda P. B. C. (2022). Artificial neural network training using metaheuristics for medical data classification: an experimental study. *Expert Systems with Applications*.

[6] Mohapatra S. K., Mohanty M. N. (2022). Big data classification with iot-based application for e-health care. *Cognitive Big Data Intelligence with a Metaheuristic Approach*.

[7] Sakalle A., Tomar P., Bhardwaj H., Acharya D., Bhardwaj A. (2021). A lstm based deep learning network for recognizing emotions using wireless brainwave driven system. *Expert Systems with Applications*.

[8] Jaya Sudha C., Sneha Y. S. (2022). Classification of medical images using deep learning to aid in adaptive big data crowdsourcing platforms. *ICT with Intelligent Applications*.

[9] Chandrashekar G., Sahin F. (2014). A survey on feature selection methods. *Computers & Electrical Engineering*.

[10] Ahmed M. R., Ali M. A., Ahmed N., Bhuiyan T. (2022). Computational intelligence approaches for prediction of chronic kidney disease. *Advances in Distributed Computing and Machine Learning*.

[11] Bhardwaj H., Sakalle A., Tiwari A., Verma M., Bhardwaj A. Breast cancer diagnosis using simultaneous feature selection and classification: a genetic programming approach.

[12] Jović A., Brkić K., Bogunović N. A Review of Feature Selection Methods with Applications.

[13] Yu J., Yu J., Almal A. A. (2007). Feature selection and molecular classification of cancer using genetic programming. *Neoplasia*.

[14] Muni D. P., Pal N. R., Das J. (2006). Genetic programming for simultaneous feature selection and classifier design. *IEEE Transactions on Systems, Man and Cybernetics, Part B (Cybernetics)*.

[15] Hashemi A., Dowlatshahi M. B., Nezamabadi-pour H. (2022). Ensemble of feature selection algorithms: a multi-criteria decision-making approach. *International Journal of Machine Learning and Cybernetics*.

[16] Bhardwaj A., Tiwari A., Varma M. V., Krishna M. R. An analysis of integration of hill climbing in crossover and mutation operation for eeg signal classification.

[17] Jain A., Pandey M., Sahu S. (2022). A deep learning-based feature extraction model for classification brain tumor. *Proceedings of Data Analytics and Management*.

[18] Lavanya D., Rani D. K. U. (2011). Analysis of feature selection with classification: breast cancer datasets. *Indian Journal of Computer Science and Engineering (IJCSE)*.

[19] Purohit A., Bhardwaj A., Tiwari A., Choudhari N. S. Removing code bloating in crossover operation in genetic programming.

The article "Genetic Programming-Based Feature Selection for Emotion Classification Using EEG Signal" was published in 2022. Journal: J Healthc Eng.

[20] Sakalle A., Tomar P., Bhardwaj H., Bhardwaj A. (2021). Emotion recognition using portable eeg device. *Communications in Computer and Information Science*.

[21] Mann H. B., Whitney D. R. (1947). On a test of whether one of two random variables is stochastically larger than the other. *The Annals of Mathematical Statistics*.

